RETRACTED

# 3D Finite Element Analysis of Seismic Response of Rigid Pile Composite Foundation with Microprobe Group

**DOI:** 10.1155/2022/6129134

**Published:** 2022-07-08

**Authors:** Li Lin, Jichao Zhang, Yadong Li, Zhuwei Rao, Zheng Sen

**Affiliations:** School of Civil Engineering, Guangzhou University, Guangzhou 510006, China

## Abstract

In order to study the seismic performance of the rigid pile composite foundation, a three-dimensional finite element analysis of the seismic response of the rigid pile composite foundation with microprobe group was proposed. The three-dimensional finite element method is used to analyze the dynamic response law of pile group rigid pile composite foundation under the action of the earthquake, especially the internal force response of the pile body. It is worth noting that when the internal force response of pile decreases significantly, the maximum internal force of the whole pile is also significantly smaller than the maximum internal force of pile foundation. However, when the pile body is located on a layered foundation and the modulus of adjacent soil layers differs greatly, the earthquake action will cause the pile body to generate a large internal force. The seismic performance of the rigid pile composite foundation is feasible, and it can be extended and applied to the similar seismic performance test of other composite foundations.

## 1. Introduction

Rigid subrigid pile composite foundation is a new and efficient foundation treatment technology, which is based on the in-depth study of the working mechanism, cushion effect, transmission characteristics, stress analysis, deformation, and bearing capacity of composite foundation at home and abroad and is widely used in engineering practice [1].

The theory and technology of composite foundation were born and advanced in the development of foundation treatment technology. Its earliest concept was proposed by Japanese scholars in the 1960s to solve the problem of the carrying capacity of the sand well foundation. Since the reform and opening up, the theory and engineering application of the composite foundation have been greatly developed in China. The definition of composite foundation and its theoretical framework based on the concept of the generalized composite foundation are put forward, and the calculation method of composite foundation bearing energy settlement has been summarized. In the aspect of theory, Gong et al. [2] put forward the concept of composite foundation and obtained the calculation method of bearing capacity at first in China; Wang et al. [3] put forward the assumption of the joint action of foundation, cushion, and pile-soil composite foundation and obtained the idea of the best share ratio; Gong et al. [4] divided the load transfer route of shallow foundation, pile foundation, and composite foundation under the load action, and through analysis, it is concluded that the essence of composite foundation is that pile and soil bear the load together directly; and Li et al. [5] finite element elastic plasticity model software of soil foundation with cushion is studied and concluded that the transfer law of friction along pile body is similar to that of pile group. In the aspect of the test, Shi et al. [6] analyzed the bearing capacity test results of rigid subrigid pile composite foundation and obtained its law; Zhou et al. [7] studied the soil arching effect and pile-soil stress ratio of composite foundation and obtained the calculation formula of pile-soil stress ratio of composite foundation; and Zhang et al. [8] analyzed the static load test of four pile large pressing plates on-site and obtained CM, and during the static load test of pile composite foundation, the mechanical characteristics of pile and soil, the failure mode, and cushion effect of CM pile composite foundation cushion are discussed. In the aspect of numerical simulation, Xing et al. [9] calculated and analyzed the different situations of composite foundation treated by rigid pile, flexible pile, and mixing pile and obtained the stress field and deformation field; Sun et al. [10] carried out numerical simulation and theoretical analysis on the settlement and bearing behavior of the rigid-flexible composite foundation and obtained that the settlement of the rigid-flexible composite foundation increased with the increase of cushion thickness, showing a nonlinear relationship; and Ma et al. [11] carried out ABAQUS three-dimensional finite element analysis on the composite foundation, and the influence of pile length on the settlement of composite foundation is obtained.

RETRACTED

As an advanced design method, the rigid subrigid pile composite foundation has a good application prospect. It will become a research hotspot in the field of civil engineering in China. Yet it is mainly statics so far. Moreover, the research on its dynamic response is still seriously lagging behind. As far as it is concerned, the main methods to study seismic problems include mainly the test method, the analytical method, and the numerical method. The shaking table test and dynamic centrifuge test have been already in application widely in the structural seismic analysis [12,13]. However, these dynamic tests still have some limitations, such as time-consuming, expensive, and limited factors. Because of its technical advantages, the finite element method can well simulate the liquefaction effect and large deformation of soil, as well as the physical characteristics of the pile-soil dynamic interaction process, which has been widely used in the structural seismic analysis [14,15].

Under the influence of the rigid pile composite foundation, the paper established the finite element calculation model, analyzed the law of dynamic stress and horizontal acceleration, and analyzed the bending moment and shear envelope of the rigid pile and the subrigid pile. The bending moment and displacement obtained from vibration table test and numerical simulation are analyzed, and the relevant research results can provide a theoretical foundation for seismic design and engineering practice of rigid one subrigid pile composite foundation.

Based on the above reasons, shaking table test and finite element numerical simulation are carried out for rigid sub-bridge pile composite foundation. The comparison between the calculation results and the test results shows that the model proposed in this paper has good accuracy and applicability. It has certain reference significance for the actual engineering design.

## 2. The Design of the Shaking Table Test

The test was carried out in the center for seismic research of Guangzhou University. It was done with the size of the shaking table being 3 m × 3 m, the frequency range 0.5–50 Hz, and maximum load 20 t. The shaking direction is three-way at six degrees of freedom, with the maximum horizontal displacement being ±100 mm, the maximum vertical displacement ±50 mm, the maximum horizontal speed ±800 mm/s, the maximum vertical speed ±500 mm/s, the maximum acceleration in horizontal direction ±1.0 g, and the maximum vertical acceleration ±2.0 g.

In the test, according to the Buckingham *π* theorem and the uniform similarity rate, the dynamic similarity coefficients of the test are determined, in which the length similarity of the structure line is 1/16, the acceleration similarity of the structure gravity is 1, and the stress similarity of the dynamic response is 1/16. The circular laminated shear model box is used in the test, which is composed of 12 layers of steel frames. Each layer of the frame can move in a horizontal direction. The diameter of the model box is 2 m, and the height is 1.44 m, as shown in Figure 1.

The pile body is proposed to be made of PMMA with a modulus of about 3.0 GPa and a density of about 1,190 kg/m^3^. The rigid pile is 800 mm long, with an outer diameter of 35 mm and an inner diameter of 30 mm. The subrigid pile is 400 mm long, with an outer diameter of 45 mm and an inner diameter of 39 mm. The clear distance between piles is 100 mm. The sand locally available and the saturated sand site in Guangzhou were selected for the test, with a soil density of 2.05 g/cm^3^; the thickness of the gravel sand cushion is 50 mm; and the sand gravel ratio is 3:7.

RETRACTED

The test pile is arranged in 4 × 4 (see Figure 2 for details). Strain gauges are arranged along the length direction of 1^#^, 2^#^, 3^#^, and 4^#^ piles with an interval of 200 mm. Acceleration sensors are arranged at the top, 2/3 away from the top, 1/3 away from the top, and the bottom of 2^#^ rigid pile and 4^#^ rigid pile. Acceleration sensors are also arranged at the top and bottom of 1^#^ subrigid pile and 3^#^ subrigid pile. In addition, acceleration sensors are placed at the bottom of the test box to monitor the output acceleration. As shown in Table 1 of the loading conditions of this test, after each set of excitations, a three-way frequency sweep is conducted with the white noise of 0.05 g.

## 3. Finite Element Simulation Software Method in the Vibration Table Test

### 3.1. Constitutive Model

#### 3.1.1. Linear Elastic Model of Pile

The stress-strain expression for the isotropic elastomer model software is as follows [16]:

(1) $$\begin{array}{c} \left\{\begin{array}{c} \varepsilon_{11}\\ \varepsilon_{22}\\ \varepsilon_{33}\\ \gamma_{12}\\ \gamma_{13}\\ \gamma_{23} \end{array}\right\}=\left[\begin{array}{cccccc} 1/E & -\nu /E & -\nu /E & 0 & 0 & 0\\ -\nu /E & 1/E & -\nu /E & 0 & 0 & 0\\ -\nu /E & -\nu /E & 1/E & 0 & 0 & 0\\ 0 & 0 & 0 & 1/G & 0 & 0\\ 0 & 0 & 0 & 0 & 1/G & 0\\ 0 & 0 & 0 & 0 & 0 & 1/G \end{array}\right]\left\{\begin{array}{c} \sigma_{11}\\ \sigma_{22}\\ \sigma_{33}\\ \sigma_{12}\\ \sigma_{13}\\ \sigma_{23} \end{array}\right\}. \end{array}$$

There are two parameters involved here, that is, modulus of elasticity and Poisson's ratio, which can vary with temperature and other field variables.

#### 3.1.2. Elastoplastic Model of Soil

Mohr–Coulomb model is used in this model.

*(1) Yield Surface.* The yield surface function of the Mohr-Coulomb model is

(2) $$\begin{array}{c} F=R_{mc}q-p\;\tan\;\phi -c=0, \end{array}$$

where *ϕ* is the inclination angle of Mohr-Coulomb yield surface on the*q*−*p* stress surface, which is called the friction angle of the material, 0° ≤ *ϕ* ≤ 90°; *c* is the cohesion of the material; *R*_*mc*_(Θ, *ϕ*) is calculated according to the following formula; it controls the shape of the yield surface in the *π* plane.

(3) $$\begin{array}{c} R_{mc}=\frac{1}{\sqrt{3}\cos\;\phi }\sin\left(\Theta +\frac{\pi }{3}\right)+\frac{1}{3}\cos\left(\Theta +\frac{\pi }{3}\right)\tan\;\phi , \end{array}$$

where Θ is the polar angle, defined as cos(3Θ)=*r*^3^/*q*^3^, and *r* is the third partial stress invariant *J*_3_.

*(2) Plastic Potential Surface.* ABAQUS uses the following continuous smooth elliptic function as the plastic potential surface, whose shape is shown in Figure 3.

(4) $$\begin{array}{c} G=\sqrt{{\left(\varepsilon c{|}_{0}\tan\;\psi \right)}^{2}+{\left(R_{mw}q\right)}^{2}}-p\;\tan\;\psi , \end{array}$$

where *ψ* is the shear expansion angle and *c|*_0_ is the initial cohesion, that is, the cohesion without plastic deformation.*ε* is the eccentricity on the meridian plane; it controls the similarity between the shape of G on the meridian and the asymptote of the function. If *ε*=0.0, the plastic potential surface will be a straight line inclined upward on the meridian plane; the default value in ABAQUS is 0.1.

RETRACTED

*R*_*mw*_(Θ, *e*, *ϕ*) controls its shape on the *π* plane, calculated by the following formula:

(5) $$\begin{array}{c} R_{mw}=\frac{4\left(1-e^{2}\right)\cos^{2}\;\Theta +{\left(2e^{2}-1\right)}^{2}}{2\left(1-e^{2}\right)\cos\;\Theta +\left(2e-1\right)\sqrt{4\left(1-e^{2}\right){\left(\cos\;\Theta \right)}^{2}+5e^{2}-4e}}R_{mc}\left(\frac{\pi }{3},\phi \right), \end{array}$$

*E* is the eccentricity on the *π* surface, which mainly controls the shape of the Θ=0 ∼*π*/3 plastic potential plane on the *π* plane. The default value is calculated by the following formula:

(6) $$\begin{array}{c} e=\frac{3-\sin\;\phi }{3+\sin\;\phi }. \end{array}$$

According to the above formula, it can be ensured that the plastic potential surface is tangent to the yield surface at the angle of *π* plane tension and compression. Of course, users can also specify the size of *e*, but its range must be 0.5 ≤ *e* ≤ 1.0. Figure 3 shows the plastic potential surfaces corresponding to different sizes.

### 3.2. Define Damping

In this paper, the implicit integration method (direct integration method) in ABAQUS is used for dynamic analysis, so the dissipation of energy can be reflected by Rayleigh damping, which is in the form of [17, 18].

(7) $$\begin{array}{c} \left[C\right]=\alpha_{R}\left[M\right]+\beta_{R}\left[K\right], \end{array}$$

where [*C*] is the damping matrix, [*K*] is the stiffness matrix, [*M*] is the mass matrix, *α*_*R*_ is the mass proportion coefficient, and*β*_*R*_ is the stiffness proportion coefficient.

The mass proportional damping coefficient and stiffness proportional damping coefficient meet the following relationship:

(8) $$\begin{array}{c} \xi_{in}=\frac{\alpha_{Ri}}{2\omega_{n}}+\frac{\beta_{Ri}\omega_{n}}{2}, \end{array}$$

where *α*_*Ri*_ is the mass proportion coefficient of the *i*-th material, *β*_*Ri*_ is the stiffness proportion coefficient of the *i*-th material, *ω*_*n*_ is the circular frequency of the *n*-th order vibration mode of the structure, and *ξ*_*in*_ is the damping ratio of the *i*-th material in the corresponding vibration mode. Taking the circular frequency and damping ratio of the first two vibration modes of the structure, two equations can be formed from the following equation, which can be obtained by combining

(9) $$\begin{array}{c} \alpha_{Ri}=\frac{2\left(\xi_{i1}/\omega_{1}-\xi_{i2}/\omega_{2}\right)}{\left(1/\omega_{1}^{2}\right)-\left(1/\omega_{2}^{2}\right)}, \end{array}$$

(10) $$\begin{array}{c} \beta_{Ri}=\frac{2\left(\xi_{i2}\omega_{2}-\xi_{i1}\omega_{1}\right)}{\omega_{2}^{2}-\omega_{1}^{2}}. \end{array}$$

RETRACTED

### 3.3. Boundary Conditions

In this paper, a series of viscous dampers are applied to each node of the artificial cutoff boundary by the spring/dashpots element directly in the preprocessing visualization interface (CAE) of ABAQUS [19,20].

According to the definition of viscous boundary, the viscous coefficient of viscous damper is

(11) $$\begin{array}{c} c=\rho c_{s}\Delta x, \end{array}$$

where *c* is the viscosity coefficient, *ρ* is the density, *c*_*s*_ is the shear wave velocity, and Δ*x* is the width of the element on both sides of the joint applied by the viscous damper.

It should be noted that for nodes on the boundary surface, only half of the width of the calculation area is involved; for nodes with different mesh widths on both sides of the node, the approximate value is

(12) $$\begin{array}{c} c=\rho c_{s}\frac{\Delta x_{1}+\Delta x_{2}}{2}. \end{array}$$

### 3.4. Establishment of the Finite Element Model Software

ABAQUS software was used for the simulation, with the elastic modulus of the pile at 3.0 GPa, Poisson's ratio 0.2, density at 1,190 kg/m^3^ in linear elastic constitutive relation, and the damping ratio at 0.05. The elastic modulus of saturated sand is 30 MPa, with Poisson's ratio at 0.22, density at 1750 kg/m^3^, internal friction angle at 30, damping ratio at 0.05, and M–C constitutive model. For the contact between pile and soil, the surface contact is defined in ABAQUS, in which the pile surface is the main control surface and the soil surface around the pile is the subordinate surface; the tangential contact model is selected as penalty friction, and the friction coefficient of pile and soil is 0.6, and the normal contact model is hard contact. The size of the cell grid plays a decisive role in the accuracy, convergence, disk space, and machine time of calculation. Generally speaking, there are the following requirements for the grid density: the grid in the area considering stress and strain should be smaller than that in the area only considering displacement; the grid should be smaller enough to capture the nonlinear effect when including nonlinearity; and if interested in the effect of wave propagation, the grid should be smaller enough to solve the wave. In this paper, an eight-node reduced integral solid element (C3D8R) is used. When the finite element method is used to study the dynamic response of an infinite medium, the artificial boundary must be introduced into the calculation model. The three-dimensional finite element model of the assembled composite foundation-shaking table test is shown in Figure 4.

RETRACTED

## 4. Analysis of Shaking Table Test and Numerical Simulation Results

### 4.1. Analysis of Acceleration-Time Curve and Fourier Spectrum

Accelerometers are arranged in the test site to monitor the acceleration response of the rigid subrigid pile composite foundation under different seismic wave excitation in a saturated sand site.

The difference in length of the rigid pile and the subrigid pile in the rigid—subrigid pile composite foundation—will definitely lead to different frequency responses. In order to study the change rule in the frequency domain, the acceleration time history curve of the measuring point is Fourier transformed, and then the change characteristics of the acceleration spectrum are analyzed. In view of the limitation of pages, this paper presents only the acceleration time curve and Fourier spectrum of the soil around the bottom of 2^#^ pile under the input of 0.2 g Taft wave, 0.4 g Taft wave, and 0.6 g Taft wave, as shown in Figure 5.

It can be seen from Figure 5 that under the three seismic wave inputs, the simulated value of acceleration time history amplitude is slightly less than the test value. It may be related to the calculation error caused by the selection of model, parameters, or boundary conditions. However, the test value and simulation value of the peak acceleration in the acceleration time history are within 30–40 s, and the shape of the test curve and simulation curve of each acceleration time history are very similar, and the peak value of the acceleration time history increases with the increase of the excitation peak value.

It can be seen from Figure 5 that under the three kinds of seismic wave input, the Fourier spectrum increases with the increase of excitation peak, and the amplitude corresponding to each frequency of the three kinds of the seismic wave increases gradually no matter the test value or the simulation value; however, the frequency distribution characteristics of the three kinds of seismic wave do not change with the increase of excitation peak, that is, the shape of the Fourier spectrum does not change with the increase of input excitation peak. The peaks of the Fourier spectrum are mainly within the frequency range of 4–7 Hz and 8–15 Hz.

RETRACTED

To sum up, it demonstrates that the modeling approach, treatment measures for some problems, and selection of calculation parameters of numerical simulation are basically consistent with the test, and the relationship between them is formed to verify the reliability of the actual earthquake reflection and reconstruction.

### 4.2. Analysis of the Acceleration Amplification Coefficient of 0.2 g Taft Wave, 0.4 g Taft Wave, and 0.6 g Taft Wave

In order to more accurately analyze the seismic amplification effect of rigid—subrigid pile composite foundation in the saturated sand site—the acceleration amplification coefficient is defined. The acceleration amplification factor is the ratio of the peak acceleration of any measuring point to the peak acceleration of the input ground motion.

It can be seen from Figure 6 that under three different excitation peak values, no matter it is the test value or the simulation value, the trend of change of the acceleration amplification coefficient of 2^#^ pile and 3^#^ pile with the direction of embedment depth is the same. In addition, the same measurement point decreases with the increase of the excitation peak. As shown in Figure6(a), under three different excitation peaks, the acceleration amplification coefficient of 2^#^ pile decreases first and then increases with the increase of embedment depth, and the acceleration amplification coefficient is less than 1. The minimum value of the acceleration amplification coefficient is ranged in the middle. It can be seen from Figure 6(b) that under the action of three different excitation peaks, the acceleration amplification coefficient of 3^#^ pile decreases with the increase of embedment depth, and the minimum value of acceleration amplification coefficient is at the bottom, which is less than 1.

It can also be observed from Figure 6 that the simulated value of acceleration amplification coefficient of 2^#^ pile and 3^#^ pile along the length direction is basically smaller than the calculated value; the simulated value of acceleration amplification coefficient of 2^#^ pile top and pile bottom is about 0.1 and 0.02, respectively, smaller than the test value; and the simulated value of acceleration amplification coefficient of 3^#^ pile top and pile bottom is about 0.02 and 0.05 smaller than the test value, respectively, which may be the acceleration response of different positions along the length direction of the pile. Different acceleration responses will affect free space. It may also be caused by the stiffness of the simulated soil being slightly greater than that of the actual soil, which makes the constraint of the soil on the pile increase. This is especially true when liquefaction occurs in the sandy soil layer in the test (due to the liquefaction criteria used in the calculation, the sandy soil is not liquefied but has been liquefied in the test).

RETRACTED

### 4.3. Strain Analysis

Before the test, the strain gauges are arranged along different positions of the pile body. Given in this paper are the test values and simulation values of the peak strain of 2^#^ pile and 3^#^ pile under the respective action of 0.2 g, 0.4 g, and 0.6 g excitation peaks of Taft wave in the saturated sand site, as shown in Figure 7.

It can be seen from Figure 7 that the peak strain of rigid pile and subrigid pile increases along with the increase of input seismic wave excitation peak value, with a gradual increase of the peak strain of the same measuring point, regardless of being either the test value or the simulation value. With the increase of the embedment depth, the change trend of the peak strain along the length direction of the pile exhibits a considerable difference.

Regardless being either the test value or the simulation value, when the excitation peak value of 2^#^ rigid pile and 3^#^ subrigid pile is 0.2 g, the minimum value of the peak value of the strain appears at the top of the pile, with little change in the peak value of the strain along the length direction of the pile. When the excitation peak value of 2^#^ rigid piles is 0.4 g and 0.6 g, the liquefaction occurs on the site, and the distribution of the peak value of the strain along the length direction is relatively abnormal, which is greater at 60 cm from the top of the pile. It may be due to the obvious stress concentration of the pile shaft caused by the sudden change of the site stiffness with the increase of the excitation peak value. 3. When the excitation peak value of 3^#^ subrigid pile is at 0.4 g and 0.6 g, the strain peak distribution along the length direction is slightly more significant than that under the excitation peak value of 0.2 g.

It can also be seen from Figure 7 that the test value of strain peak value is very close to the absolute value of simulation value, and the overall transformation trend is also very consistent. The test results are slightly larger than the simulation results, and the numerical simulation curve is relatively smooth. It may be related to the limitations of the test; the test results can only get part of the time strain; and the finite simulation can better solve this problem, and the strain during the full range of time can be obtained from the simulation results.

## 5. Conclusion

Based on the shaking table test and finite element simulation of the composite foundation with rigid and subrigid piles in saturated sandy soil carried out in this paper, it can be concluded after the analysis that:

1. Under the three kinds of seismic wave input, the simulation value of acceleration time history amplitude is slightly smaller than the test value; with the increase of excitation peak value, the amplitude corresponding to each frequency of the three kinds of the seismic wave increases gradually, regardless of the test value or the simulation value, but the shape of the Fourier spectrum does not change with the increase of input excitation peak value.
2. Under the action of three kinds of excitation peaks, the amplification coefficient of pile acceleration changes in accordance with the direction of embedment depth. In addition, the same measurement point decreases with the increase of excitation peaks.
3. The test value of strain peak is close to the simulation value in absolute quantity, and the overall transformation trend is also very consistent. The test results are slightly larger than the simulation results, and the numerical simulation curve is relatively smooth.
4. Under the action of the three kinds of seismic waves, the acceleration response strength of the rigid pile first decreases and then increases with the increase of embedment depth; the strength of acceleration response of the subrigid pile gradually decreases along with the increase of the embedment depth, while along with the increase of excitation peak, the distribution change of the strain peak along the length direction of the pile body becomes increasingly significant of which, abnormality appears at the peak strain distribution of the rigid pile along the length of the pile body, which is the weak part in terms of earthquake resistance.

RETRACTED

## Figures and Tables

**Figure 1:** Model box.

**Figure 2:** Layout of test piles: (a) plan view and (b) sectional view.

**Figure 3:** Plastic potential surface in Mohr–Coulomb model.

**Figure 4:** 3D finite element model.

**Figure 5:** Comparison of acceleration-time curve and Fourier spectrum test value and simulation value at the bottom of 2^#^ pile: (a) under the action of seismic wave of 0.2 g Taft, (b) under the action of seismic wave of 0.4 g Taft, and (c) under the action of seismic wave of 0.6 g Taft.

**Figure 6:** Comparison of test and simulation values of acceleration amplification coefficient of (a) 2^#^ pile and (b) 3^#^ pile.

**Figure 7:** Test and simulation values of peak strain of 2^#^ pile and 3^#^ pile: (a) test value of peak strain of 2^#^ pile and 3^#^ pile and (b) simulation value of peak strain of 2^#^ pile and 3^#^ pile.

**Table 1:** The loading conditions of this test.

Type of input seismic wave	Peak acceleration (g)	Test site
Taft wave	0.2	Saturated sand
Taft wave	0.4	Saturated sand
Taft wave	0.6	Saturated sand

RETRACTED

## Data Availability

The data used to support the findings of this study are available from the corresponding author upon request.

## References

[1] CAO (2018). The study of working principle and the suitability of the CM composite foundation soil. the degree of master of engineering in science. *EEE/ASME Transactions on Mechatronics*.

[2] Gong X. (1992). *Summary of Composite Foundation Theory, the third foundation treatment Symposium of foundation treatment*.

[3] Wang C., Guo X. (1996). Interaction principle of foundation cushion composite foundation. *Journal of Civil Engineering*.

[4] Gong X.. (2007). Theory and engineering application of generalized composite foundation. *Journal of geotechnical engineering*.

[5] Jianjun L. I., Liang R. W., Bai X. (2009). Finite element analysis of load transfer characteristics of cement soil pile composite foundation. *Journal of Taiyuan University of Technology*.

[6] Shi Q. (2005). Analysis of bearing capacity test results of CM pile composite foundation. *Geotechnical engineering technology*.

[7] Zhao W., Yang G. (2011). Study on soil arching effect and pile-soil stress ratio of composite foundation. *Journal of Civil Engineering*.

[8] Jixin U., Zhang H., Zhou Y. (2015). Field test and Study on pile-soil stress ratio and cushion effect of CM pile composite foundation. *Geotechnical mechanics*.

[9] Xing Z., Chen X. (2013). Study on Mechanical Properties and Finite Element Analysis of Composite Foundation. *Journal of Sound and Vibration*.

[10] Sun L.. (2009). *Nonlinear Finite Element Analysis of Rigid Flexible Pile Composite Foundation*.

[11] Rui M. A. (2016). Analysis on the influence of long short pile composite foundation on foundation settlement in loess area. *Journal of Liaoning Institute of Technology*.

[12] Sheng G. (2013). Seismic performance analysis of piles in rigid pile composite foundation. *Geotechnical mechanics*.

[13] Zhong R., Huang M. (2014). Centrifugal test of seismic response of caisson pile composite foundation. *Geotechnical mechanics*.

[14] Lu J., Elgamal A., Yan L., Law K. H., Conte J. P (2011). Large-scale numerical modeling in geotechnical earthquake engineering. *International Journal of Geomechanics*.

[15] Ni K., GAO W. (2013). Numerical simulation of shaking table test for seismic performance of pile foundation and rigid composite foundation. *Building Science*.

[16] Kang F. E. I., Zhang J. (2010). *Application of ABAQUS in Geotechnical Engineering*.

[17] Yin Z., Zhu H., Xu G. (1994). Deformation and numerical simulation of interface between soil and structural materials. *Journal of geotechnical engineering*.

RETRACTED

[18] Zhang Ga, Zhang J. (1994). Elastoplastic constitutive model of soil structure interface for interaction between single pile and foundation. *Journal of geotechnical engineering*.

[19] Zong L. I. (2019). Dynamic Interaction Analysis of Soil Underground Ground Structure.

[20] Li Y., Jingshan B. O., Sun Q. (2017). Realization and application of viscous boundary conditions in ABAQUS. *Construction Technology*.

